The article "Application of Higher Education Management in Colleges and Universities by Deep Learning" was retracted in 2023. Reasons: signs of a paper mill; suspected computer-generated content; unreliable results or conclusions; concerns about the data.

# Application of Higher Education Management in Colleges and Universities by Deep Learning

**DOI:** 10.1155/2022/7295198

**Published:** 2022-08-10

**Authors:** Ge Yao

**Affiliations:** School of International Education, Anshan Normal University, Anshan 114005, Liaoning, China

## Abstract

The development of artificial intelligence (AI) has brought great convenience to people and has been widely used in the field of education. To monitor the classroom status of college students in real time and achieve the purpose of balanced distribution of educational resources, the facial expression recognition (FER) algorithm is applied to the management of higher education in universities. Firstly, the convolutional neural network (CNN) is studied in depth, and secondly, the process and method of FER are explored in detail, and an adaptive FER algorithm based on the differential convolutional neural network (DCNN) is constructed. Finally, the algorithm is applied to the CK + database and the BU-4DFE database. The results manifest that the designed algorithm has an accuracy of 99.02% for keyframe detection in the CK + database and 98.35% for the BU-4DFE database. The algorithm has a high accuracy of keyframe detection for both expression databases. It has a good effect on the automatic detection of keyframes of expression sequences and can reach a level similar to that of manual frame selection. Compared with the existing algorithms, the proposed method still has higher advantages. It can effectively eliminate the interference of individual differences and environmental noise on FER. Experiments reveal that the proposed FER algorithm DCNN-based has a good recognition effect and is suitable for monitoring students' classroom status. This research has certain reference significance for the application of AI in higher education management in colleges and universities.

## 1. Introduction

In recent years, the progress of artificial intelligence (AI) has greatly changed people's work and lifestyle, and intelligence has appeared in various fields, bringing great convenience to people. Education is considered to be one of the most important topics for a family. With the emphasis on education by the country and the family, the number of students is increasing year by year, followed by a serious imbalance between the number of teachers and the number of students. Teachers cannot take into account the classroom status of all students, while ensuring the quality of education. The level of higher education management affects students' own development to a certain extent. Good education management can create the best learning and growth space for students. AI-assisted education can help to achieve education fairness and improve the level of education management [1].

The article "Application of Higher Education Management in Colleges and Universities by Deep Learning" was retracted in 2023. Reasons: signs of a paper mill; suspected computer-generated content; unreliable results or conclusions; concerns about the data.

Face recognition is complex and diverse. It has become an urgent problem to be solved in the field of facial expression recognition (FER) to study how to improve the accuracy of FER and the generalization ability of the model in practical applications and to enhance the superiority of the algorithm. At present, the application of AI in education around the world is mainly divided into adaptive learning education, virtual assistant, expert system, business intelligence, etc., and this research proposes a FER algorithm on account of differential convolutional neural network (DCNN) and applies it to the education management system of the universities [2]. Facebook proposed the DeepFace algorithm for FER under deep learning (DL) at the Conference on Computer Vision and Pattern Recognition (CVPR) in 2014. The algorithm first performs face detection, annotates the detected face with 67 base points, constructs a 3D model of the face, aligns the nonfrontal faces, and finally inputs it into the network for recognition. The algorithm eventually achieved 97.35% accuracy on the Labeled Faces in the Wild (LFW) dataset [3]. In 2015, Google published the FaceNed algorithm on CVPR, which combines convolutional neural network (CNN) with triple loss and maps faces to Euclidean space. The similarity between the mapped face vectors is calculated, and the accuracy reaches 99.63% on the LFW dataset and 95.12% on the YouTube face dataset, which is nearly 30% higher than before [4]. In 2018, Tencent proposed a FER algorithm CosFace under DL based on large-interval cosine loss at CVPR. This algorithm converts the loss function into a cosine loss function by normalizing the feature vector and weight vector. On this basis of this, a cosine edge value is introduced to further maximize the decision boundary of the learned feature in the angle space. The algorithm not only achieves a high recognition rate in LFW but also achieves an accuracy of 98% on the MegaFace dataset [5]. In 2021, some scholars proposed a method of combining the two-dimensional principal component analysis (PCA) method and the improved linear discriminant analysis method and applied it to the face recognition technology, thereby improving the recognition rate of the algorithm [6]. Although there are many studies on FER algorithms and good results have been achieved, there are relatively few studies on the application of FER algorithms to higher education management in colleges and universities. Therefore, this research applies it to universities' higher education management to monitor the classroom status of students in real time. By grasping the facial expressions of students, judging learning status, and providing feedback for teaching, the educational resources can be fully utilized.

The article "Application of Higher Education Management in Colleges and Universities by Deep Learning" was retracted in 2023. Reasons: signs of a paper mill; suspected computer-generated content; unreliable results or conclusions; concerns about the data.

The purpose is to identify students' classroom facial expressions and learning emotions, monitor students' classroom status, and improve the level of education management. The DCNN is integrated with the FER algorithm, and the algorithm is applied to the education management system of colleges and universities. First, the process and method of CNN and FER are deeply studied. Then, the DCNN-based FER algorithm is constructed on this basis. At last, the expression database is trained by the experimental training method, and the recognition effect of the designed algorithm is further verified. It has certain reference significance for the application of AI in higher education management in colleges.

## 2. Materials and Methods

### 2.1. Convolutional Neural Network

Compared with traditional neural network (NN), CNN has three important characteristics: local connectivity, weight sharing, and pooling, which improves the robustness of the model to noise and better solves the computational difficulty caused by too many parameters in high-dimensional input [7].

Research in the field of biological vision has found that people's perception of the outside world is generally from a local to a whole. The adjacent pixels are more closely connected, and the pixels that are far away are almost irrelevant [8]. Inspired by this, the neurons in the convolutional layer of CNN do not need to be connected to all neurons, but only need to be connected to some neurons in the neighborhood, and then the local information is integrated to obtain the global information. The application of local connectivity strategies can effectively reduce the number of parameters that need to be learned in the network [9]. The schematic diagram of full and local connectivity is shown in Figure 1.

In two-dimensional (2D) images, the statistical characteristics of all local regions are similar, and the same convolution kernel can be used for feature extraction. However, the same kind of convolution kernel can only extract the same kind of features, so multiple convolution kernels can be applied in actual training to improve feature diversity [10]. The weight-sharing strategy can not only reduce the number of parameters for network training and enhance the generalization ability of the network but also use different convolution kernels to map a variety of feature maps, thereby extracting rich image information [11].

After the convolution operation, the training parameters can be significantly reduced, but the dimension of the extracted features is still very high, which may cause the classifier to face the curse of dimensionality and overfitting [12]. To solve the above problems, it is proposed to add a pooling layer after the convolutional layer, that is, after the convolution operation is completed, downsampling is performed, and the features of different local positions are aggregated and counted. Specific pooling methods include max pooling, mean pooling, and random pooling. [13]. The pooling strategy can effectively reduce the number of parameters, prevent overfitting, and enable the model to achieve scaling invariance of image transformation.

The article "Application of Higher Education Management in Colleges and Universities by Deep Learning" was retracted in 2023. Reasons: signs of a paper mill; suspected computer-generated content; unreliable results or conclusions; concerns about the data.

Influenced by traditional NN, CNN also adopts a similar hierarchical structure. Each layer consists of multiple 2D feature maps, each of which contains multiple independent neurons. Many CNN variants have emerged in recent years, but their basic components are very similar. The classic LeNet-5 is taken as an example, and its network structure is displayed in Figure 2.

LeNet-5 is mainly composed of convolutional layers, pooling layers, and fully connected layers. The functions of convolutional layers like feature extractors aim to learn feature representations of input images. Convolutional layers consist of multiple convolution kernels to obtain local information at different locations on the image [14]. The functions of convolutional layer, pooling layer, and fully connected layer can be used to extract face recognition features and facial expression information. The convolution kernel performs convolution calculation on the coverage area through the feature map output by the previous layer, to obtain different feature maps and learn different types of features. The specific convolution process is that each convolution kernel is connected to the local area of the feature map of the previous layer, and each parameter of the convolution kernel is multiplied by the corresponding local pixel value and the bias is added, that is, the 2D convolution is completed. Then, through the activation function calculation, multiple feature maps are obtained as outputs and passed to the next layer of neurons. The equation of the convolutional layer is as follows:

(1) $$\begin{array}{c} y_{j}^{p}=\theta \left(\sum_{i=1}^{N_{i}^{p-1}}w_{i,j}⊗x_{j}^{p-1}+b_{j}^{p}\right),\;j=1,2,\ldots ,M, \end{array}$$

where *p* layer expresses the current layer, *p* − 1 layer indicates the previous layer, *yp*/*j* is the *j* th feature map of the current layer, *w*_*i*,*j*_ stands for the convolution kernel between the *j* th feature map of the current layer and the *i* th feature map of the previous layer, *xp* − 1/*j* illustrates the *j* th feature map of the previous layer, and *bp*/*j* signifies the bias value of the *j* th feature in the current layer. *N*_*i*_^*p*−1^ is the number of feature maps connecting the *j* th feature map of the current layer to the previous layer. *M* refers to the total number of feature maps of the current layer, *θ*(·) represents the activation function, and ⊗ means the convolution operation [15].

The article "Application of Higher Education Management in Colleges and Universities by Deep Learning" was retracted in 2023. Reasons: signs of a paper mill; suspected computer-generated content; unreliable results or conclusions; concerns about the data.

The pooling layer is usually placed between two convolutional layers to reduce the dimension of the feature map output by the convolutional layer, reduce network parameters and computational complexity, improve feature robustness, and avoid overfitting. The pooling layer reduces the number of feature maps while maintaining the number of feature maps, which not only preserves the salient features of the original feature maps but also reduces the model's sensitivity to transformations such as translation, scaling, and rotation [16]. Pooling calculates the value of each local area of the feature map and replaces the original feature output with the statistical feature value, to achieve the purpose of scaling the feature map. Assuming that the size of the sampling window is *n∗n*, after one downsampling, the size of the feature map becomes the original 1/*n*^2^. The expression of the pooling layer is demonstrated as

(2) $$\begin{array}{c} y_{j}^{p}=\theta \left(\varphi_{j}^{p}\text{down}\left(y_{j}^{p-1}\right)+b_{j}^{p}\right),\;j=1,2,\ldots ,M, \end{array}$$

where *yp*/*j* denotes the *j* th feature map of the current layer, *φp*/*j* shows the multiplicative bias value of the *j* th feature map of the current layer, *y*_*j*_^*p*−1^ manifests the *j* th feature map of the previous layer, *bp*/*j* indicates the additive bias value, and down (·) represents the downsampling function.

The neurons of the fully connected layer are all interconnected with the neurons of the previous layer, and the 2D feature map is mapped to a one-dimensional feature vector with a preset length. All features are synthesized through this fully connected operation and output as the final feature is extracted. Because of its fully connected feature, the parameters of this layer account for about 90% of the entire CNN, and these parameters have an important impact on the classification effect of the model [17]. The large number of parameters contained in the fully connected layer also brings difficulties to network training. Researchers began to explore ways to replace the fully connected layer or reduce the number of connections. GoogleNet used sparse connections to replace the fully connected layer to reduce the amount of computation, and achieved good results [18]. The output of the fully connected layer is illustrated as follows:

(3) $$\begin{array}{c} h_{x,b}\left(x\right)=\theta \left(\omega^{T}\left(x\right)+b\right), \end{array}$$

where *h*_*x*,*b*_(*x*) means the output value of the fully connected layer, *x* illustrates the input feature vector, *ω* is the weight vector, *b* refers to the bias value, and *θ*(·) represents the activation function.

The article "Application of Higher Education Management in Colleges and Universities by Deep Learning" was retracted in 2023. Reasons: signs of a paper mill; suspected computer-generated content; unreliable results or conclusions; concerns about the data.

### 2.2. The Process of FER

FER refers to analyzing a given face image or image sequence to find unique information that can characterize facial expressions, and the image is then identified as a specific expression category. The ultimate goal of automatic facial expression recognition (AFER) is to enable computers to have the ability to understand human emotions and respond intelligently, thereby enhancing the experience of the human-computer interaction (HCI) [19]. The FER algorithm is usually completed in three steps, as displayed in Figure 3.

In Figure 3, the FER algorithm firstly performs face detection and image preprocessing on the original database. That is, the use of computer detection and positioning of face regions, and further alignment and normalization processing, to avoid the influence of expression-independent factors such as complex backgrounds, occlusions, and light intensity. After that, the expression features of the face image are extracted, and the quality of the extracted features plays a decisive role in the effect of expression recognition, so it is also the most critical step. Besides, because most feature extractions have the problem of dimensionality disaster, feature dimensionality reduction is also required. In the end, the expression features are sent to a suitable classifier to complete the expression classification [20, 21].

In recent years, more researchers have begun to use DL methods for expression recognition. Compared with traditional methods, its advantage lies in that it can train models in an end-to-end manner and automatically learn features related to facial expressions without manual production. It not only reduces manual intervention and algorithm complexity but also extracts features that are deeper and more relevant to expressions [22].

The facial expression database is limited by the collection conditions. Usually, in addition to the human face, there are interferences such as complex backgrounds in the image. If the original image is directly input to extract expression features, it will bring a large negative effect to the recognition results [23]. Hence, to reduce the influence of irrelevant factors as much as possible, face detection and positioning should be performed on the original image, and the background interference in the detection frame should be minimized, to obtain pure facial image data that can accurately represent the expression information. The two most commonly used algorithms are face detection using the AdaBoost algorithm and the DL-based face detection algorithm. The core idea of the AdaBoost algorithm is to extract different features from the same training set to train multiple weak classifiers. After many iterations, the weak classifiers with excellent performance in the training process are selected to construct strong classifiers. These strong classifiers are combined in a certain structure to form a cascaded classifier with a cascade structure, to achieve an ideal detection result. Although this method greatly improves the detection speed, it has higher requirements on posture, background, angle, and illumination. The DL-based face detection algorithm solves the problem that the traditional method is sensitive to illumination, background, angle, etc., to a certain extent. FacenessNet is used for face detection. Five kinds of facial features are extracted by training five CNNs, and the local features are integrated to determine the face region. This method can utilize both global and local feature information to improve detection accuracy [24–26].

The article "Application of Higher Education Management in Colleges and Universities by Deep Learning" was retracted in 2023. Reasons: signs of a paper mill; suspected computer-generated content; unreliable results or conclusions; concerns about the data.

### 2.3. FER Algorithm by Using DCNN

The two-stage adaptive expression recognition algorithm framework based on DCNN is proposed, and the algorithm flow is demonstrated in Figure 4.

In Figure 4, the facial expression sequence is sent to the two-class CNN, and the keyframes of the output sequence are detected, that is, the neutral expression frame and the peak expression frame. The keyframe selection strategy is based on the SoftMax value corresponding to each frame. The keyframes are sent to DCNN, the differential depth features between the keyframes are extracted, and the expression category corresponding to the sample sequence is considered output.

The SoftMax function is a generalization of the logistic function. SoftMax is used in the multiclassification process. It maps the outputs of multiple neurons into an interval, which can be understood as a probability, so it can be used for multiclassification. The output result of the SoftMax classifier is the probability value of classifying the input image into each class. If it is a K-class classifier, the output is a K-dimensional vector. Each dimension represents the probability of an input sample being assigned to that classification, and the elements in the vector sum to 1 [27]. For the training set composed of *m* samples and its labels, it is denoted as {(*x*^(1)^, *y*^(1)^),…, (*x*^(*m*)^, *y*^(*m*)^)}, *y*^(*i*)^ ∈ {1,2,…, *k*}. The *k* estimated probabilities of each sample are as follows:

(4) $$\begin{array}{c} h_{\theta }\left(x^{\left(i\right)}\right)=\left[\begin{array}{c} p\left(y^{\left(i\right)}=1|x^{\left(i\right)};\theta \right)\\ p\left(y^{\left(i\right)}=2|x^{\left(i\right)};\theta \right)\\ \cdots \\ p\left(y^{\left(i\right)}=k|x^{\left(i\right)};\theta \right) \end{array}\right]=\frac{1}{\sum_{j=1}^{k}e^{\theta_{j}^{T}x^{\left(i\right)}}}\left[\begin{array}{c} e^{\theta_{1}^{T}x^{\left(i\right)}}\\ e^{\theta_{2}^{T}x^{\left(i\right)}}\\ \cdots \\ e^{\theta_{k}^{T}x^{\left(i\right)}} \end{array}\right], \end{array}$$

where *k* is the number of classification categories; *θ*_1_, *θ*_2_,…, *θ*_*k*_ ∈ *R*^*n*+1^ are network model parameters; 1/∑_*j*=1_^*k*^*e*^*θ*_*j*_^*T*^*x*^(*i*)^^ means that the results are normalized, and the sum of the probabilities of all categories is 1.

The article "Application of Higher Education Management in Colleges and Universities by Deep Learning" was retracted in 2023. Reasons: signs of a paper mill; suspected computer-generated content; unreliable results or conclusions; concerns about the data.

The SoftMax function accumulates the *k* possible categories, that is, the probability for classifying the sample *x* into category *j* by the SoftMax classifier is obtained as

(5) $$\begin{array}{c} p\left(y^{\left(i\right)}=j|x^{\left(i\right)};\theta \right)=\frac{e^{\theta_{j}^{T}x^{\left(i\right)}}}{\sum_{l=1}^{k}e^{\theta_{l}^{T}x^{\left(i\right)}}}. \end{array}$$

The category corresponding to the maximum probability is the classification category of *x*. To complete the network training, it needs to use the gradient descent method to minimize the loss function of SoftMax. The loss function is exhibited as

(6) $$\begin{array}{c} L_{s}=-\frac{1}{m}\left[\sum_{i=1}^{m}\log\frac{e^{\theta^{\left(i\right)}}}{\sum_{l=1}^{k}e^{\theta_{l}^{T}x^{\left(i\right)}}}\right]. \end{array}$$

In practical applications, to prevent any parameter *θ* from being 0, weight decay is usually added to the loss function. The larger the loss function, the smaller the probability that the classifier will classify correctly. The best performance is achieved by successive iterative computation of the minimum value of the loss function to obtain the global optimal solution [28].

In the process of DNCC training, the depth features of the keyframes of the expression sequence are first extracted. The feature *a*^*N*^ is extracted from the neutral expression frame by the convolutional layer of N-net, and the feature *a*^*F*^ is extracted from the peak expression frame by the convolutional layer of F-net. After that, the calculation process of the FC1 layer of the two branch networks is shown as follows:

(7) $$\begin{array}{c} \left\{\begin{array}{c} Z^{N}=W^{N}a^{N}+b^{N},C^{N}=f\left(Z^{N}\right),\\ Z^{F}=W^{F}a^{F}+b^{F},C^{F}=f\left(Z^{F}\right), \end{array}\right. \end{array}$$

where *W*^*N*^ and *W*^*F*^ express the weight parameters of the network; *b*^*N*^ and *b*^*F*^ stand for the bias values; *f*(·) means the activation function; *C*^*N*^ and *C*^*F*^ are the network output value of N-net and F-net, respectively. Next, the differential depth features between keyframes are calculated. The output values *C*^*N*^ and *C*^*F*^ of N-net and F-net are, respectively, sent to the differential layer to complete the calculation and extraction of the differential depth feature *a*^diff^, which is expressed as

(8) $$\begin{array}{c} a^{\text{diff}}=C^{F}-C^{N}=f\left(Z^{F}\right)-f\left(Z^{N}\right). \end{array}$$

The differential depth feature is sent to the fully connected layer FC2, FC3, and SoftMax classification layer to complete the expression recognition. In the training phase, all weight layers of DCNN use the original parameters of the Visual Geometry Group (VGG) 16 model to complete parameter initialization, and all weight values are set to a trainable state. Moreover, at the beginning of training, the parameter values of the two branch networks N-net and F-net at the corresponding positions are set to be the same. Based on the above equations, the weight update equation of the first weight layer is as follows:

(9) $$\begin{array}{c} W^{l+}=W^{l}-\eta \frac{\partial J\left(W,b\right)}{\partial W},\\ b^{l+}=b^{l}-\eta \frac{\partial J\left(W,b\right)}{\partial b}. \end{array}$$

In equation (9), *η* is the learning rate. Then the gradient calculation of the FC1 layer is expressed as follows:

(10) $$\begin{array}{c} \left\{\begin{array}{c} \frac{\partial J\left(W,b\right)}{\partial W^{N}}=\frac{\partial J\left(W,b\right)}{\partial Z^{\text{FC}2}}\frac{\partial Z^{\text{FC}2}}{\partial a^{\text{diff}}}\frac{\partial a^{\text{diff}}}{\partial Z^{N}}\frac{\partial Z^{N}}{\partial W^{N}}=-{\left(W^{\text{FC}2}\right)}^{T}\delta^{\text{FC}2}f^{\prime }\left(Z^{N}\right){\left(a^{N}\right)}^{T},\\ \frac{\partial J\left(W,b\right)}{\partial W^{F}}=\frac{\partial J\left(W,b\right)}{\partial Z^{\text{FC}2}}\frac{\partial Z^{\text{FC}2}}{\partial a^{\text{diff}}}\frac{\partial a^{\text{diff}}}{\partial Z^{F}}\frac{\partial Z^{F}}{\partial W^{F}}={\left(W^{\text{FC}2}\right)}^{T}\delta^{\text{FC}2}f^{\prime }\left(Z^{F}\right){\left(a^{F}\right)}^{T},\\ \frac{\partial J\left(W,b\right)}{\partial b^{N}}=\frac{\partial J\left(W,b\right)}{\partial Z^{\text{FC}2}}\frac{\partial Z^{\text{FC}2}}{\partial a^{\text{diff}}}\frac{\partial a^{\text{diff}}}{\partial Z^{N}}\frac{\partial Z^{N}}{\partial b^{N}}=-{\left(W^{\text{FC}2}\right)}^{T}\delta^{\text{FC}2}f^{\prime }\left(Z^{N}\right),\\ \frac{\partial J\left(W,b\right)}{\partial b^{F}}=\frac{\partial J\left(W,b\right)}{\partial Z^{\text{FC}2}}\frac{\partial Z^{\text{FC}2}}{\partial a^{\text{diff}}}\frac{\partial a^{\text{diff}}}{\partial Z^{F}}\frac{\partial Z^{F}}{\partial b^{F}}={\left(W^{\text{FC}2}\right)}^{T}\delta^{\text{FC}2}f^{\prime }\left(Z^{F}\right), \end{array}\right. \end{array}$$

where *W*^FC2^ is the weight vector of the FC2 layer and *δ*^FC2^ = *∂Z*^FC2^/*∂a*^diff^ is the residual value of the FC2 layer.

The article "Application of Higher Education Management in Colleges and Universities by Deep Learning" was retracted in 2023. Reasons: signs of a paper mill; suspected computer-generated content; unreliable results or conclusions; concerns about the data.

In this experiment, the facial expression database consisting of facial expression dynamic image sequences is selected: CK+ and BU-4DFE. The CK+ expression database is collected by 123 college students aged 18–30 years by shooting videos of facial expressions under laboratory conditions, and they are all frontal shots. Among them, the proportion of women is 65%, and the data includes African-Americans, Asians, and South Americans. The library consists of 7 types of expressions: angry, disgusted, scared, happy, sad, surprised, and contemptuous, with a total of 593 image sequences, of which only 327 sequences have expression category labels. The first frame of each sequence is a neutral expression image, and the last frame is a peak expression image corresponding to the emotion label. The length of the whole sequence varies from 10 to 60 frames. All images are 640*∗*490 pixels, most of them are grayscale images, and some are color images. The BU-4DFE expression database collects facial expression data of Asian, African, Latino, European, and other ethnic groups, including 43 males and 58 females, a total of 101 persons. Each sample object in the library contains six basic types of expressions: angry, disgusted, afraid, happy, sad, and surprised. Expressions are collected and organized in the form of video sequences, including a total of 606 expression sample sequences. Among them, most of the sequences recorded the process from no expression to the peak of expression to the end of the expression, and a few sequences only recorded the process from the peak of expression to the end of the expression, and the average length of the sequence was 100 frames. All images in this library have a resolution of 1040*∗*1329 pixels, and all faces are taken from the front, which is very suitable for analyzing 2D facial expressions.

In order not to affect the effect of the expression features extracted in the subsequent experiments, the accuracy of expression recognition is reduced. Therefore, face detection is performed on the image to determine whether there is a face, as well as the specific position and size of the face, and then a pure face area image is obtained by clipping, and the facial expression image is uniformly normalized to a size of 256*∗*256.

## 3. Results and Discussion

### 3.1. Expression Recognition Performance of DCNN

The two databases selected in this experiment are tested by the method of fivefold cross-validation, that is, the data is split into five parts, four of which are selected for training each time, and the remaining one is used for testing. The sets do not cross each other, a total of five experiments are carried out, and the average of the results of the five experiments is taken as the end result. The key frame detection is performed by the SoftMax function, and the accuracy of the keyframe detection of the binary CNN on the database CK+ and BU-4DFE is finally measured, as demonstrated in Figure 5.

The article "Application of Higher Education Management in Colleges and Universities by Deep Learning" was retracted in 2023. Reasons: signs of a paper mill; suspected computer-generated content; unreliable results or conclusions; concerns about the data.

Figure 5 signifies that the accuracy for the CK+ database is stable at 99.02%, and the accuracy for the BU-4DFE database is stable at 98.35%. To further verify its performance, the automatically extracted keyframes and the manually selected keyframes are sent to DCNN at the same time. The results of expression recognition are output and compared, as shown in Figure 6.

In Figure 6, on the CK+ database, the recognition rate of manual frame selection is 97.5%, and the recognition rate of automatic frame selection is 95.4%. The result of the FER based on automatic frame selection is only 2.1% lower than that of manual frame selection. On the BU-4DFE database, the recognition rate of manual frame selection is 79.4%, and the recognition rate of automatic frame selection is 77.4%, which is only a decrease of 2%. The above experiments can fully prove that the proposed automatic detection method of expression sequence keyframes has a good effect, and can even reach a level similar to that of manual frame selection.

### 3.2. Comparison of Experimental Results

For a more scientific evaluation of the performance of the proposed DCNN-based FER algorithm, it is compared with existing advanced technical methods, including neutral-subtracted (NES), pairwise conditional random forests (PCRF), CNN + LandmarkE, Pre-CNN, deep peak-neutral difference (DPND), and DPND + deep representations of peak (DPND + DRP). To clearly compare the performance of different algorithms, the result analysis is expressed in Figure 7 and Table 1.

In Figure 7 and Table 1, the proposed method achieves a recognition rate of 96.7% on CK+ and 77.4% on BU-4DFE. The recognition rate is higher than that of other algorithms. The results of the proposed method on BU-4DFE are better than other algorithms, and even based on automatic frame selection, the accuracy on CK+ is still 3.8% higher than that of DPND. The experimental results strongly demonstrate the superiority of the end-to-end model. Further, DCNN (manual frame selection) has a 1.6% increase in the accuracy of CK+ compared to pre-CNN without any data augmentation, which proves that the proposed method can effectively eliminate the interference of individual differences and environmental noise on FER.

The article "Application of Higher Education Management in Colleges and Universities by Deep Learning" was retracted in 2023. Reasons: signs of a paper mill; suspected computer-generated content; unreliable results or conclusions; concerns about the data.

## 4. Conclusion

To better identify students' classroom emotions, monitor students' status during class, and improve education management, this research applies the DCNN-based FER algorithm to the education management system of colleges. First, the CNN is deeply explored, then the process and method of FER are studied, and the FER algorithm on the strength of DCNN is constructed. At last, it is verified by experiments that the proposed FER algorithm by DCNN has a good recognition effect and is suitable for students' classroom status monitoring. The experimental result reveals that the accuracy of the keyframe detection of the database is 99.02%, and for the BU-4DFE database is 98.35%. And the results of the FER based on automatic frame selection only decreased by 1.3% compared with manual frame selection and only decreased by 2% on the BU-4DFE database. Moreover, compared with the existing algorithms, the proposed method still has higher benefits, which can effectively eliminate the interference of individual differences and environmental noise on FER. For emotion recognition, by collecting the facial expressions of students in the classroom, it is found that many expressions have relatively small amplitudes. Therefore, it is not accurate enough to perform emotion recognition by using the feature of facial expression. In the follow-up, various emotional expression information such as gestures, speech, and physiological signals will be considered to be added to explore the emotional computing model of multifeature fusion. This research has certain reference significance for the application of AI in higher education management in colleges and universities. The innovation is that a two-stage adaptive expression recognition algorithm based on differential CNN is proposed. Compared with other algorithms, the proposed algorithm has a good recognition effect and high superiority and can effectively eliminate the interference caused by individual differences and environmental noise on FER.

## Figures and Tables

**Figure 1:** Schematic diagram of fully and local connectivity. (a) A schematic diagram of full connectivity; (b) a schematic diagram of local connectivity.

**Figure 2:** Schematic diagram of the LeNet-5 structure.

**Figure 3:** Steps of the FER algorithm.

**Figure 4:** Flowchart of the algorithm.

**Figure 5:** The accuracy of the keyframe detection of binary CNN on CK+/BU-4DFE.

**Figure 6:** The recognition rate of six types of expressions by DCNN on CK+/BU-4DFE.

The article "Application of Higher Education Management in Colleges and Universities by Deep Learning" was retracted in 2023. Reasons: signs of a paper mill; suspected computer-generated content; unreliable results or conclusions; concerns about the data.

**Figure 7:** Comparative experimental results of different algorithms in CK+/BU-4DFE.

**Table 1:** Comparison of different algorithms in CK+/BU-4DFE.

Technology and methods	CK+	BU-4DFE
NES	96	74.8
PCRF	96.4	76.1
CNN + LandmarkE	93.1	75.9
Pre-CNN	96.8	76.4
DPND	92.9	76.6
DPND + DRP	94.4	78.4
DCNN (manually)	98	79.4
DCNN (automatically)	96.7	77.4

## Data Availability

The experimental data used to support the findings of this study are available from the corresponding author upon request.
